This article has been retracted.

# Repression of CRNDE enhances the anti‐tumour activity of CD8 + T cells against oral squamous cell carcinoma through regulating miR‐545‐5p and TIM‐3

**DOI:** 10.1111/jcmm.16909

**Published:** 2021-11-02

**Authors:** Yilong Ai, Siyuan Wu, Hai Gao, Haigang Wei, Zhe Tang, Xia Li, Chen Zou

**Affiliations:** ^1^ School of Stomatology and Medicine Foshan Stomatological Hospital Foshan University Foshan China; ^2^ Department of Prosthodontics Stomatological Hospital Southern Medical University Guangzhou China

**Keywords:** CRNDE, immune response, miR‐545‐5p, OSCC, TIM‐3

## Abstract

Immunotherapy has been identified a promising treatment of cancers, including Oral squamous cell carcinoma (OSCC). CRNDE is highly overexpressed in various cancers. Many lncRNAs have been reported in CD8 T lymphocytes. Little is investigated about their effects in the functions of CD8 + T cells in OSCC. Currently, the influence of lncRNA CRNDE on the function of CD8 + T cells in OSCC progression was investigated. Here, CRNDE was obviously elevated and negatively correlated with IFN‐γ production in tumour‐infiltrating CD8 + T cells isolated from OSCC patients. CRNDE can exhibit a crucial role in activating CD8 + T‐cell exhaustion. Mechanistically, CRNDE specifically sponged miR‐545‐5p to induce T‐cell immunoglobulin and mucin domain‐3 (TIM‐3), thus contributing to CD8 + T‐cell exhaustion. The function of miR‐545‐5p on T‐cell function remains poorly known. TIM‐3 is a significant immune checkpoint, and it inhibits cancer immunity. TIM‐3 can demonstrate an important role in CD8 + T‐cell exhaustion. In summary, loss of CRNDE could induce miR‐545‐5p and inhibit TIM3 expression, thus significantly activated the anti‐tumour effect of CD8 + T cells.

## 1 INTRODUCTION

Oral squamous cell carcinoma (OSCC) is a frequent head and neck malignant tumour. It almost occupies approximately 3% in clinical cancer cases.^1^ Recently, in spite of great progress is made in OSCC, overall 5‐year survival rate still remains unsatisfactory with a 5‐year survival of 40%–50%.^2^, ^3^ Due to the poor early diagnosis, OSCC is usually identified at the advanced stages. Smoking, consumption of alcohol and betel quid chewing are potential risk factors contributing to OSCC progression.^4^ Chemoradiotherapy and radiotherapy photodynamic therapy are the treatment of OSCC with serious side effects due to non‐specific cell death.^5^, ^6^ Hence, it is urgent to improve the treatment of OSCC.

Tumour‐infiltrating lymphocytes (TILs) are well described in cancers.^7^, ^8^ In OSCC, the presence of TILs is a positive indicator for OSCC.^9^ In addition, the immune infiltrate of tumours has various lymphocytes, in which, T cells are a kind of crucial cell types.^10^, ^11^ An enrichment of T‐cell infiltrates indicates favourable clinical outcome in cancers.^12^ In addition, it has been shown that OSCC patients with elevated ratio of CD8^+^ T cells have a better outcome.^13^, ^14^, ^15^

Noncoding RNAs are classified into microRNAs (less than 200nt) and lncRNAs (more than 200nt, lncRNA).^16^, ^17^ Dysregulated lncRNAs and microRNAs expression in cancer may serve as predictors for various cancer outcomes.^18^, ^19^ LncRNAs can function via regulating mRNA translation through competitively combining with miRNAs.^20^ LncRNA CRNDE can contribute a lot to colorectal cancer via regulating miR‐181a‐5p.^21^ CRNDE can promote the development of hepatocellular carcinoma via regulating miR‐217 and MAPK1.^22^ Nevertheless, the effect of CRNDE in immune response of OSCC remains elusive. Meanwhile, by using bioinformatics analysis, CRNDE has many known and potential targets. The function of miR‐545‐5p on T‐cell function remains unknown. Here, we investigated the correlation between CRNDE and miR‐545‐5p in T‐cell function in OSCC progression.

In our current work, CRNDE was aberrantly increased in OSCC and promoted the malignant phenotypes of OSCC cells. CRNDE promoted CD8 + T‐cell exhaustion. Notably, miR‐545‐5p was predicted as the potential target of CRNDE using bioinformatics tools. Up‐regulation of CRNDE was negatively associated with miR‐545‐5p level. TIM3 could act as a downstream target of miR‐545‐5p. Our study depicted a lncRNA CRNDE/miR‐545‐5p/TIM‐3 regulatory network in the activity of CD8 + T cells.

## 2 METHODS AND MATERIALS

### 2.1 Tissue samples

Fifteen paired OSCC tissues and adjacent non‐tumorous tissues were acquired from patients at Stomatological Hospital, Southern Medical University. The fifteen tumour samples utilized had been confirmed as OSCC specimens by three pathologists. Non‐cancerous tissues were more than 2cm away from clinically identified tumour tissues. Non‐cancerous tissues were submitted for histopathological confirmation. Before the surgery, no patients received any radiotherapy or chemotherapy. Written informed consent was obtained. Tissues were frozen in liquid nitrogen and maintained at −80℃. Fifteen healthy donors and fifteen OSCC patients were involved for blood samples at Stomatological Hospital, Southern Medical University to isolate peripheral or tissue‐infiltration lymphocytes. This work obtained the approval from the Ethical Committee of Stomatological Hospital, Southern Medical University (ECR‐20180106).

### 2.2 Cell culture

Normal human oral keratinocyte (NHOK) and OSCC cells (SCC9, SCC‐25, SCC‐15, FaDu and TU‐183) were purchased from ATCC (Manassas, VA, USA). Cells were incubated in DMEM with 10% FBS and 1% penicillin/streptomycin. A humidified atmosphere at 37℃ with 5% CO_2_ was used.

### 2.3 Lymphocyte isolation and culture

Peripheral blood lymphocytes (PBLs) were isolated using Ficoll density gradient centrifugation. In brief, dissociated cells from OSCC tissue sections were filtered through a 75 mm cell strainer and separated via Ficoll centrifugation. The mononuclear cells were resuspended in DMEM medium added with 10% FBS. CD8 + T cells were added with TAKARA GT‐T551 medium (Takara, Japan) containing human IL‐2.

### 2.4 Plasmid construction and lentivirus infection

In order to induce CRNDE expression, the ORF sequence of PCAT6 was cloned into pTracer‐CMV2 vector (Jingmai BioTech). OSCC cells were transfected with 2 μg CRNDE‐OE or empty control vector by Lipofectamine 3000 (Thermo Fisher Scientific). To down‐regulate CRNDE, small hairpin sequence was cloned into pLKO.1 plasmid with the vectors employed as control. Subsequently, PSPAX2‐PMD2G system was carried out to package the lentivirus.

### 2.5 RNA extraction and quantitative real‐time PCR

To do quantitative detection of CRNDE, miR‐545‐5p and TIM‐3, total RNA was extracted using TRIzol. Then, via carrying out a Reverse Transcription Kit (Takara), isolated RNA was reversely transcribed to cDNA. Afterwards, a SYBR‐Green PCR Master Mix kit (Takara) on ABI Prism 7,900 Sequence Detection System (Applied Biosystems) was used to do qRT‐PCR analysis. Then, gene expression was calculated by 2^−ΔΔCt^ approach. All the primers were shown in Table 1.

**TABLE 1:** Primers for real‐time PCR

Targets	Forward (5′−3′)	Reverse (5′−3′)
GAPDH	GGGAGCCAAAAGGGTCAT	GAGTCCTTCCACGATACCAA
CRNDE	TGGATGCTGTCAGCTAAGTTCAC	TTCCAGTGGCATCCTCCTTATC
miR−545‐5p	TCAGTAAATGTTTATTAGATGA	GTGCAGGGTCCGAGGTATTC
TIM−3	AAGACCTTGGACTCTCAAACTCG	CCTGGTAAATGAGCCGTTGTTTT
U6	TCCGATCGTGAAGCGTTC	GTGCAGGGTCCGAGGT

### 2.6 Western blotting analysis

Total protein was extracted, and BCA method was carried out to test protein concentration. Then, protein was separated on 10% SDS‐PAGE. After finishing electrophoresis, protein was transferred to PVDF membrane. Then, the membrane was subjected to 5% skim milk. The membranes were processed with primary antibodies against GAPDH and TIM‐3 (Abcam). The membrane was incubated with horseradish‐peroxidase‐bound secondary antibodies for 2 h. Then, the membrane was visualized by an ECL system.

### 2.7 CCK‐8 assay

Cell Counting Kit‐8 (CCK‐8) (Dojindo, Kumamoto, Japan) was employed to test cell proliferation. Cells were loaded into 96‐well plates and incubated for a whole night. CCK‐8 reagents were added to the cells for various time points. Spectra Max M2 was employed to measure OD values at 450 nm.

### 2.8 EdU analysis

BeyoClick™ EdU Cell Proliferation Kit was used to test cell proliferation. Transfected cells were incubated with 10 µM EdU for 2 h. Then, cells were fixed for 30 min in 4% PFA before stained by DAPI for 30 min. Finally, cells were imaged using an inverted microscope.

### 2.9 Transwell assay

For evaluating cell migration, cells were seeded to the upper chambers of Transwell chambers added with medium added with 10% FBS. 24 h later, a cotton swab was employed to wipe off non‐migratory cells. Migratory cells were fixed and stained. To test cell invasion, the specific step was pre‐coated with matrigel (Corning) in the upper chambers. Afterwards, process of abovementioned procedures was followed.

### 2.10 Luciferase reporter assay

Sequences of WT or MUT of CRNDE promoter was sub‐cloned into pGL3‐basic vector. Then, these plasmids were co‐transfected into OSCC cells with miR‐545‐5p mimics. Sequences of WT or MUT of TIM‐3 promoter were sub‐cloned into pGL3‐basic vector. Afterwards, these plasmids were co‐transfected into OSCC cells with miR‐545‐5p mimics or inhibitors. Dual‐Luciferase reporter assay system was used to evaluate luciferase activities.

### 2.11 RIP assay

Magna RNA‐binding protein immunoprecipitation (RIP) kit was used to carry out RIP assay. 3 μg anti‐Ago2 antibody (Abcam) and anti‐IgG antibody were added at 4℃ with cell lysates overnight. Then, the mixture was incubated with 25 μL protein A/G beads. Finally, precipitated RNAs were obtained to do qRT‐PCR analysis.

### 2.12 Cytolysis activity assay

Oral squamous cell carcinoma cells were employed as the target cells. Prior to the assay, OSCC cells were radiolabelled with [methyl‐ 3 H] thymidine to a concentration of 5μ Ci/ml for 24h. CD8 + T cells transfected with CRNDE‐OE or sh‐CRNDE were incubated with labelled OSCC cells for a whole night.

### 2.13 Generation of OSCC‐specific CD8 + T cells

Naïve CD8 + T cells from peripheral blood mononuclear cells PBMCs, density gradients separated by Ficoll (GE Healthcare) were purified using the EasySep TM Human CD8 + T Cell Enrichment Kit. Generation of OSCC‐specific CD8 + T cells were stimulated with 1 μg/ml CD3 mAb and 5 μg/ml CD28 mAb in RPMI 1,640 medium with 10% foetal bovine serum, 20 ng/ml human rIL‐2, 50 U/ml penicillin and 50 mg/Ml streptomycin. Then, dendritic cells were differentiated from adherent monocytes in RPMI 1640 medium. IL‐4 (50 ng/ml) and GM‐CSF (100 ng/ml) were then added. One week later, the obtained DCs were incubated with heat‐shocked OSCC cells to obtain antigen‐loaded DCs (APCs). Naïve CD8 + T cells were subjected to lentiviral infection of CRNDE‐OE or shRNA. These treated naïve T cells were incubated with APCs for 3 days to obtain tumour antigen‐specific CD8 + T cells.

### 2.14 OSCC mouse model

To carry out the xenograft OSCC mouse model, 2 × 10^6^ SCC‐15 cells were mixed with Matrigel 1:7 in 100 µl and subcutaneously inoculated in the right groin of (BABL/c nude, male, 6‐week‐old). APC‐stimulated naïve CD8 + T cells (pretreated with CRNDE‐OE or shRNA, 1 × 10^7^ cells each mouse) were injected into the caudal vein to reconstitute the human immune system. Tumours were extracted 22 days later after CD8 + T cell transfer and the tumour tissues were isolated for the further assays. All animal experiments were based on the Guide for the Care and Use of Laboratory Animals of the National Institutes of Health.

### 2.15 Immunochemistry

Tissues from the mice were fixed using 4% paraformaldehyde. After dehydration and embedded, the samples were sliced into 5 μm thickness. The slices were stained with Ki‐67 antibody at 4℃. After Sav‐HRP conjugates incubation, sections were incubated with DAB substrate and observed using a microscopy (Zeiss, German). The counterparts were stained by H&E.

### 2.16 Flow cytometry

To test the frequencies of IFN‐γ+ and TNF‐α in CD8 + T cells, tumour cells were fixed, permeabilized and stained with anti‐CD8‐APC, anti‐IFNγ‐PE or anti‐TNF‐α‐FITC (BD Biosciences). Staining with fluorophore‐conjugated secondary antibodies was followed for flow cytometry analysis.

### 2.17 Immunofluorescent staining

After air‐dried, tissue sections were washed using PBS and blocked by 10% normal serum blocking solution‐species the same as the secondary antibody. Afterwards, the sections were incubated by primary antibodies for anti‐CD8 (1:100, eBioscience) for 20 h at 4℃ and followed by Alexa Fluor 488 conjugated secondary antibodies (eBioscience). After stained using DAPI, sections were examined with using confocal microscope (Leica Microsystems).

### 2.18 Statistical analysis

Data were presented as means ± SD. Data were analysed using SPSS version 17.0 and Prism 6.0. One‐way analysis of variance with multiple comparisons using Dunnett's test was utilized to do multiple comparison. Pearson's correlation test was used to assess the association among CRNDE, miR‐545‐5p and TIM‐3 in OSCC. *p *< 0.05 was considered to be significant.

## 3 RESULTS

### 3.1 Overexpression of CRNDE indicated the exhaustion of CD8 + T lymphocytes in OSCC

To explore the role of CRNDE in OSCC, CRNDE expression in OSCC tissues was determined using qRT‐PCR analysis. The relationship between clinicopathological features and CRNDE expression level was analysed and shown in Table 2. Overexpression of CRNDE in fifteen pair of OSCC tissues was observed (Figure 1A). The expression of CRNDE in OSCC patients at stage Ⅳ was significantly increased compared to stages Ⅰ, Ⅱ and Ⅲ as shown in Figure 1B. In addition, in Figure 1C, CRNDE was increased in OSCC cell lines. CRNDE expression was obviously increased in tumour‐infiltrating T cells in comparison with the peripheral blood T cells from OSCC patients and healthy controls (Figure 1D). Furthermore, a negative correlation was observed between CRNDE expression and the ratio of IFN‐γ+ CD8 + T cells in tumour‐infiltrating CD8 + T cells of OSCC patients as shown in Figure 1E. These suggested the overexpression of CRNDE was closely related to CD8 + T cells.

**TABLE 2:** Clinicopathological relevance analysis of CRNDE in OSCC patients

Feather	Patients	CRNDE		
		Low	High	*p* value
Cases	15	6	9	
Age, years				
<60	6	3	3	0.525
≥60	9	4	5	
Gender				
Male	8	3	5	0.366
Female	7	4	3	
T stage				
T1‐T2	6	3	3	0.443
T3‐T4	9	5	4	
N stage				
N0	5	3	2	0.205
N+	10	6	4	
Stage				
Ⅰ,Ⅱ,Ⅲ	5	4	1	**0.012**
Ⅳ	10	3	7	
Nodal Invasion				
Positive	3	1	2	0.349
Negative	12	5	7	
Differentiation				
Differentiated	13	7	6	0.562
Undifferentiated	2	1	1	

Bold value indicates *p* value less than 0.05.

**FIGURE 1:** Up‐regulation of CRNDE was correlated with CD8 + T cells in OSCC. (A) Expression of CRNDE in the tumour tissues of OSCC patients (*n* = 15) and the healthy tissues (*n* = 15). (B) The expression of CRNDE in OSCC patients at various stages. (C) The expression of CRNDE in different types of OSCC (SCC9, SCC‐25, SCC‐15, FaDu and TU‐183) cells and NHOK cells using qRT‐PCR analysis. (D) Relatively level of CRNDE in tumour‐infiltrating CD8 T cells (TIL‐T), the peripheral blood CD8 T cells of OSCC patients (PBL‐T) and healthy controls (PBL‐C). (E) Pearson's correlation of CRNDE expression and the percentage of IFN‐γ + CD8 T cells in the tumour‐infiltrating CD8 T cells were analysed. (*n* = 15). *, *p* < 0.05; ***, *p* < 0.001

### 3.2 Overexpression of CRNDE aggravated the progression of OSCC

Then gain‐of‐function assays were performed in SCC‐15 and SCC‐25 cells. CRNDE was effectively elevated in OSCC cells (Figure 2A). Cell viability was significantly enhanced by CRNDE‐OE as shown in Figure 2B. In addition, SCC‐15 and SCC‐25 cell migration and invasion were increased by CRNDE overexpression (Figure 2C, D). To examine whether the increased CRNDE expression induced by CRNDE‐OE in SCC‐15 and SCC‐25 cells may impact the cytotoxicity of CD8 + T cells, we co‐cultured CD8 + T cells (effector cells) with OSCC cells (target cells) which overexpressed CRNDE. As displayed in Figure 2E, F, CRNDE‐OE significantly reduced the cytotoxicity of the CD8 + T cells against OSCC cells. These indicated CRNDE overexpression repressed the cytotoxicity of CD8 + T cells.

**FIGURE 2:** Overexpression of CRNDE aggravated the progression of OSCC. (A) qRT‐PCR revealed that CRNDE was effectively increased in SCC‐15 and SCC‐25 cells using CRNDE‐OE. (B) CCK‐8 showed cell viability were enhanced by CRNDE‐OE. (C and D) Transwell assay was used to test cell migration and invasion. (E and F) Cytolysis activity of CD8 + T cells against OSCC cells was detected after cell transfection. *, *p* < 0.05

### 3.3 **CRNDE sponged miR‐545‐5p**.

Moreover, miR‐545‐5p was predicted as the target for CRNDE. Putative binding sites between CRNDE and miR‐545‐5p were exhibited in Figure 3A. In Figure 3B, C, luciferase activity was reduced in OSCC cells co‐transfected with CRNDE‐WT and miR‐545‐5p mimics. In Figure 3D, E, RIP assay was used to evaluate the condition between CRNDE and miR‐545‐5p. We observed that CRNDE and miR‐545‐5p were greatly presented in the Ago2 protein complex. Expression of miR‐545‐5p was reduced in OSCC tissues and cells as indicated using qRT‐PCR analysis (Figure 3F, G). In Figure 3H, Pearson's correlation displayed miR‐545‐5p expression was positively correlated with IFN‐γ + CD8 + T cells. These data implied CRNDE could sponge miR‐545‐5p.

**FIGURE 3:** CRNDE sponged miR‐545‐5p. (A) The putative binding sites between CRNDE and miR‐545‐5p. (B and C) Luciferase activity was evaluated in OSCC cells co‐transfected with CRNDE‐WT or CRNDE‐MUT reporter and miR‐545‐5p mimics. (D and E) RIP assay was carried out to assess the binding condition between CRNDE and miR‐545‐5p. (F) Expression of miR‐545‐5p in the tumour tissues of OSCC patients (*n* = 15) and the healthy tissues (*n* = 15). (G) The expression of miR‐545‐5p in different types of OSCC (SCC9, SCC‐25, SCC‐15, FaDu and TU‐183) cells and NHOK cells using qRT‐PCR analysis. (H) Pearson's correlation of miR‐545‐5p expression and the percentage of IFN‐γ + CD8 + T cells. (*n* = 15). *, *p* < 0.05

### 3.4 **Inhibition of miR‐545‐5p contributed to the progression of OSCC**.

CRNDE shRNA and miR‐545‐5p inhibitors were transfected into SCC‐15 and SCC‐25 cells to evaluate the effect of miR‐545‐5p in OSCC progression. Figure 4A, B proved miR‐545‐5p expression in OSCC cells was successfully reduced by miR‐545‐5p inhibitors, which was increased by CRNDE shRNA. SCC‐15 and SCC‐25 cell proliferation was triggered by loss of miR‐545‐5p (Figure 4C, D). Moreover, OSCC cell migration and invasion were increased after miR‐545‐5p inhibitors were used Figure 4E, F. Transfecting OSCC cells with CRNDE shRNA was sufficient to promote the cytotoxicity of the CD8 + T cells against OSCC cells, while down‐regulating miR‐545‐5p in CRNDE shRNA‐transfected OSCC cells reversed these effects (Figure 4G, 4H **)**. These implied loss of miR‐545‐5p contributed to OSCC progression via repressing immune responses.

**FIGURE 4:** Inhibitors of miR‐545‐5p exacerbated the progression of OSCC. (A and B) qRT‐PCR analysis of miR‐545‐5p in SCC‐15 and SCC‐25 cells transfected with CRNDE‐shRNA and miR‐545‐5p inhibitors. (C and D) EdU assay was carried out to assess OSCC cell proliferation. Scale bar = 100 µm. (E and F) Cell migration and invasion capacity. (G and H) Cytolysis activity of CD8 + T cells against OSCC cells was tested after transfection. *, *p* < 0.05

### 3.5 **TIM‐3 acted as a target of miR‐545‐5p**.

TIM‐3 was predicted as the target for miR‐545‐5p, due to its important roles in immune responses. The binding sites between TIM‐3and miR‐545‐5p were exhibited in Figure 5A. In Figure 5B, C, luciferase activity was reduced in OSCC cells co‐transfected with CRNDE‐WT and miR‐545‐5p mimics while induced by miR‐545‐5p inhibitors. In Figure 5D, E, TIM‐3 expression was repressed by miR‐545‐5p mimics in OSCC cells. TIM‐3 mRNA expression in OSCC cells was successfully reduced by loss of CRNDE, which could be reversed by miR‐545‐5p inhibitors (Figure 5F). In Figure 5G, Pearson's correlation displayed miR‐545‐5p expression was negatively correlated with CRNDE. For another, In Figure 5H, a positive correlation between CRNDE and TIM‐3 expression. These indicated TIM‐3 acted as a target of miR‐545‐5p.

**FIGURE 5:** miR‐545‐5p targeted TIM‐3. (A) The putative binding sites between TIM‐3 and miR‐545‐5p. (B and C) Luciferase activity was evaluated in OSCC cells co‐transfected with TIM‐3‐WT or TIM‐3‐MUT reporter and miR‐545‐5p mimics or inhibitors. (D and E) TIM‐3 expression in OSCC cells transfected with miR‐545‐5p mimics. (F) qRT‐PCR analysis of TIM3 in SCC‐15 and SCC‐25 cells transfected with CRNDE‐shRNA and miR‐545‐5p inhibitors (G) Pearson's correlation of miR‐545‐5p and CRNDE expression in the tumour‐infiltrating CD8 + T cells. (H) Pearson's correlation of TIM‐3 and CRNDE expression in tumour‐infiltrating CD8 + T cells was analysed. *, *p* < 0.05

### 3.6 **Overexpression of CRNDE in naïve CD8 + T cells increased OSCC growth in vivo**.

To further investigate the role of immune cell‐expressed CRNDE in the tumorgenesis of OSCC, 2 × 10^6^ SCC‐15 cells were mixed with Matrigel 1:7 in 100 µl and subcutaneously inoculated in the right groin of the nude mice. We overexpressed CRNDE in naïve CD8 + T cells isolated from the peripheral blood of healthy donors, which were then incubated with OSCC antigen‐loaded DCs to obtain antigen‐specific CD8 + T cells. Then, these CD8 + T cells were transferred into OSCC tumour‐bearing nude mice. CRNDE‐OE‐treated CD8 + T cells markedly increased tumour growth in Figure 6A. Then, we sacrificed the moribund OSCC mice to evaluate the tumour microenvironment. HE staining analysis was carried out, and Ki‐67 staining was stronger in CRNDE‐OE‐treated group as displayed in Figure 6B. The percentage of IFN‐γ‐ and TNF‐α‐producing CD8^+^ T cells was significantly decreased by CRNDE‐OE treatment in Figure 6C, D. These results indicated CRNDE greatly repressed the immune response in OSCC in vivo.

**FIGURE 6:** CRNDE impaired the immune response in OSCC. CRNDE was overexpressed in naïve CD8 + T cells isolated from the peripheral blood of healthy donors, which were then incubated with OSCC antigen‐loaded DCs to obtain antigen‐specific CD8 + T cells. (A) Tumour volume in a time‐dependent manner. (B) Immunohistochemical staining for Ki‐67 (Scale bar = 50 µm) and HE staining analysis (Scale bar = 20 µm). (C) Quantification of the frequency of IFN‐γ and CD8 + T cells in tumour sections by flow cytometry. (D) Quantification of the frequency of TNF‐α and CD8+ T cells in tumour sections by flow cytometry. *, *p* < 0.05

### 3.7 **Knockdown of CRNDE in naïve CD8 + T cells activated the immune response in OSCC in vivo via regulating miR‐545‐5p and TIM‐3**.

Subsequently, to confirm whether the detailed mechanism of CRNDE involving miR‐545‐5p and TIM‐3 in OSCC, we inhibited CRNDE in naïve CD8 + T cells isolated from the peripheral blood of healthy donors and then they were incubated with OSCC antigen‐loaded DCs to obtain antigen‐specific CD8 + T cells. These CD8 + T cells were transferred into OSCC tumour‐bearing nude mice. CRNDE shRNA‐treated CD8 + T cells markedly decreased tumour growth in Figure 7A. Representative confocal microscopy images of CD8 staining with DAPI in tumour tissues was exhibited, and we observed that loss of CRNDE induced CD8 + T‐cell ratios as shown in Figure 7B. Frequency of IFN‐γ‐ and TNF‐α‐producing CD8^+^ T cells was significantly increased by loss of CRNDE in Figure 7C, D. CRNDE and TIM‐3 were down‐regulated by sh‐CRNDE while miR‐545‐5p was strongly increased (Figure 7E, F, G, H). Finally, in Figure 7I, summarization of CRNDE/miR‐545‐5p/TIM‐3 axis in OSCC progression involving CD8 + T‐cell function was manifested. These indicated knockdown of CRNDE activated the immune response in OSCC in vivo by modulating miR‐545‐5p and TIM‐3.

**FIGURE 7:** Loss of CRNDE activated the immune response in OSCC. CRNDE was silenced in naïve CD8 + T cells isolated from the peripheral blood of healthy donors and then incubated with OSCC antigen‐loaded DCs to obtain antigen‐specific CD8 + T cells. (A) Tumour volume. (B) Confocal analysis staining of CD8 + T cells. Scale bar = 100 µm. (C) Quantification of the frequency of IFN‐γ and CD8 + T cells in tumour sections by flow cytometry. (D) Quantification of the frequency of TNF‐α and CD8 + T cells in tumour sections. (E) CRNDE expression in the tumour tissues. (F) miR‐545‐5p expression in the tumour tissues. (G and H) TIM‐3 expression in the tumour tissues. (I) Summarization of CRNDE/miR‐545‐5p/TIM‐3 axis in OSCC progression. *, *p* < 0.05

## 4 DISCUSSION

Due to its functions in cancer progression, CRNDE has been considered as a significant tumour promoter.^23^, ^24^, ^25^ In addition, lncRNA CRNDE can regulate cell growth in OSCC.^26^ Here, the effect of CRNDE on the malignant behaviours was confirmed. We found overexpression of CRNDE enhanced CD8 + T‐cell exhaustion and reduced the cytolysis activity against OSCC via regulating miR‐545‐5p and TIM‐3. These data indicated an effective therapeutic target for OSCC immunotherapy.

LncRNA can participate in cell proliferation and immune responses in various cancers.^27^ For instance, lncRNA UCA1 can promote immune escape and reduce apoptosis in gastric cancer.^28^ OSTN‐AS1 can represent an immune‐related prognostic marker for breast cancer.^29^ Changes in immune surveillance also indicate crucial hallmarks of OSCC, and our study investigated the biological role of CRNDE in the immune escape of OSCC. CRNDE was increased in OSCC tissues and cells. Up‐regulation of CRNDE contributed to OSCC progression via inducing CD8 + T cells exhaustion. Up‐regulation of CRNDE in PBLs from OSCC patients suggests it as a diagnostic biomarker of OSCC. Downstream effects of targeting CRNDE in OSCC development needs more investigation.

The interaction between CRNDE and miR‐545‐5p was well explored. Our findings unravelled a novel regulatory system in the anti‐tumour activity of CD8 + T cells. miR‐545‐5p is associated with the tumorigenesis of various cancers. For example, miR‐545 can repress the development of lung cancer through the inactivation of Wnt/β‐catenin and targeting ZEB2.^30^ miR‐545 represses pancreatic ductal adenocarcinoma via inhibiting RIG‐I.^31^ Radiotherapy can inhibit tumour‐specific recruitment of regulator T cells by inducing miR‐545 in lung cancer cells.^32^ In our work, we confirmed the direct correlation between miR‐545‐5p and CRNDE. We proved that inhibitors reversed the effect of sh‐CRNDE on OSCC progression involving CD8 + T‐cell function. In our future study, a coculture system using CD8 + T cells and OSCC cells is required to explore the effect of CRNDE in OSCC progression.

Then, we found that through targeting TIM‐3, miR‐545‐5p exhibited immune regulation function in OSCC. TIM‐3 has been recognized as a crucial participant in cancer immunotherapy, especially in the dysfunctional phenotypes of CD8 + T cells in cancer.^33^ Tim‐3 exerts a role in regulating immune responses in different cancers and Tim‐3 has been identified as an effective target for cancer immunotherapy.^34^ Up‐regulation of miR‐545‐5p greatly reduced TIM‐3 expression and a positive correlation between TIM‐3 and CRNDE was displayed in OSCC tissues. Subsequently, we proved that loss of CRNDE significantly activated the immune responses of OSCC via regulating miR‐545‐5p and TIM‐3. Knocking down CRNDE in T cells reduced OSCC tumour growth, which might exhibit a decreased expression of CRNDE in cancer cells. In our future study, in vitro study to survey how CRNDE knockdown T cells interact with OSCC cells is warranted.

In conclusion, CRNDE was involved in the immune escape of OSCC via modulating miR‐545‐5p and TIM‐3. These findings might offer a theoretical basis for effective immunotherapy to improve the outcomes in OSCC.

## CONFLICTS OF INTEREST

The authors confirm that there are no conflicts of interest.

## AUTHOR CONTRIBUTIONS

**Yilong Ai:** Investigation (equal); Validation (equal); Visualization (equal); Writing‐original draft (equal). **Siyuan Wu:** Data curation (equal); Investigation (equal); Visualization (equal). **Haigang Wei:** Formal analysis (equal); Investigation (equal); Methodology (equal); Software (equal). **Zhe Tang:** Data curation (equal); Validation (equal); Visualization (equal). **Xia Li:** Conceptualization (equal); Project administration (equal); Writing‐review and editing (equal). **Chen Zou:** Conceptualization (equal); Resources (equal); Writing‐review & editing (equal). **Hai Gao:** Data curation (equal); Investigation (equal); Writing‐review and editing (equal).

## Data Availability

The data that support the findings of this study are available from the corresponding author upon reasonable request.
